The article "Methylation-mediated silencing of microRNA-211 promotes cell growth and epithelial to mesenchymal transition through activation of the AKT/β-catenin pathway in GBM" was retracted in 2026. Reasons: plagiarized images; duplicated images; overlap with other authors' work.

# Methylation-mediated silencing of microRNA-211 promotes cell growth and epithelial to mesenchymal transition through activation of the AKT/β-catenin pathway in GBM

**DOI:** 10.18632/oncotarget.15531

**Published:** 2017-02-20

**Authors:** Weidong Li, Xiaobo Miao, Lingling Liu, Yue Zhang, Xuejun Jin, Xiaojun Luo, Hai Gao, Xubin Deng

**Affiliations:** ^1^ Affiliated Cancer Hospital of Guangzhou Medical University, Guangzhou, China; ^2^ Department of Radiation and Chemotherapy Oncology, Ningbo No.2 Hospital, Ningbo, China; ^3^ Department of Hematology, The Third Affiliated Hospital of Sun Yat-sen University, Guangzhou, China; ^4^ Department of Radiation Oncology, The First Affiliated Hospital, Zhengzhou University, Zhengzhou, China; ^5^ Traditional Chinese Medicine-Integrated Hospital of Southern Medical University, Guangzhou, China; ^6^ Xiamen Hospital of Traditional Chinese Medicine, Xiamen, China; ^7^ Xiamen Hospital Affiliated to Fujian University of Traditional Chinese Medicine, Xiamen, China

**Keywords:** glioblastoma, miR-211, HMGA2, EZH2, epithelial to mesenchymal transition

## Abstract

Aberrant expression of miR-211 has frequently been reported in cancer studies; however, its role in glioblastoma multiforme (GBM) has not been examined in detail. We investigated the function and the underlying mechanism of miR-211 in GBM. We revealed that miR-211 was downregulated in GBM tissues and cell lines. Restoration of miR-211 inhibited GBM cell growth and invasion both *in vitro* and *in vivo*. The epithelial to mesenchymal transition (EMT) phenotype was reversed when miR-211 expression was restored. HMGA2 was identified as a down-stream target of miR-211. MiR-211 had an inhibitory effect on AKT/β-catenin signaling, which was reversed by HMGA2 overexpression or miR-211 restoration. In addition, miR-211 was transcriptionally repressed by EZH2-induced H3K27 trimethylation and promoter methylation. Overall, our findings revealed miR-211 as a tumor suppressor in GBM and mir-211 may be a potential therapeutic target for GBM patients.

## INTRODUCTION

Glioblastoma multiforme (GBM), the most common brain cancer in adults, is notorious for its diffuse invasion and resistance to treatment [1, 2]. Although major therapeutic improvements were made by combining neurosurgery, chemotherapy, and radiotherapy, the prognosis and survival rate for patients with GBM is poor [3]. The 5 year survival rate of GBM patients is less than 5% [4]. Thus, there is an urgent need to find new strategies for the treatment of GBM.

MicroRNAs (miRNAs), a class of endogenous non-coding RNAs of 19–25 nucleotides in length, negatively regulate protein expression through complimentary base pairing with the 3′-untranslated region (3′-UTR) of target mRNAs [5, 6]. MiRNAs not only contribute to diverse biological processes, but also to the progression and metastasis of human cancers [7, 8]. Abnormal expression of miRNAs often leads to GBM progression.

Epigenetic silencing by DNA methylation is one of many mechanisms of miRNA suppression in human cancer. Enhancer of zeste homolog 2 (EZH2), a methyltransferase and the core catalytic element of the polycomb repressive complex 2 (PRC2), can induce the genome-wide histone H3 lysine 27 trimethylation (H3K27me3) and acts as an oncogene via the repression of tumor suppressor genes in human cancers [9, 10]. Recent studies have well documented that EZH2 could suppress miRNAs expression through inducing H3K27me3 on the miRNAs promoter region [11].

Previous studies have demonstrated that miR-211 plays different roles across different cancers. Mir-211 is suggested to function as a tumor suppressor in ovarian cancer [12], hepatocellular carcinoma [13], triple-negative breast cancer [14] and pancreatic cancer [15]. However, miR-211 promotes cell proliferation in head and neck cancer [16]. In oral squamous cell carcinoma, miR-211 is associated with poor patient survival and enhances the oncogenicity of carcinogen-induced oral carcinoma [17]. These results suggest that miR-211′s function may be different depending on the tumor subtype. To date, the expression and clinical significance of miR-211 in GBM is still poorly understood.

The aim of our study is to explore the role of miR-211 in GBM progression. In the present study, we detected miR-211 expression in GBM tissues and cell lines. In addition, we explored the molecular mechanisms underlying the suppressive function of miR-211 in GBM. Furthermore, we revealed that miR-211 downregulation was mediated by EZH2-induced methylation.

## RESULTS

### miR-211 expression was downregulated in GBM cell lines and tissues

We first examined the expression of miR-211 in GBM tissues and cell lines with the use of qRT-PCR. The results demonstrated that miR-211 expression was significantly downregulated in all four GBM cell lines when compared to normal brain cells (NBC) (Figure 1A). Cell line U87, which had the lowest expression of miR-211, was chosen for further study. In addition, we revealed that miR-211 expression was significantly decreased in GBM tissues versus normal brain tissues, as determined by RT-PCR and in situ hybridization assays (Figure 1B and 1C). In a large cohort of 98 GBM patients, the Kaplan-Meier analysis revealed a significant decrease in overall survival time between the high miR-211 group and low miR-211 group (Figure 1D).

**Figure 1:** miR-211 expression was downregulated in GBM cell lines and tissues **A**. miR-211 expression was downregulated in GBM cell lines, when compared with normal brain cells (NBC). **B**. miR-211 expression was significantly decreased in GBM tissues versus corresponding non-tumor tissues, as determined by RT-PCR. **C**. An in situ hybridization assay was performed to examine the expression of miR-211 in GBM tissues and non-tumor tissues. **D**. GBM patients with high miR-211 expression had longer overall survival time than those with low miR-211 expression.

### Restoration of miR-211 inhibited GBM cell growth and invasion

We then asked whether miR-211 restoration affected cell growth and invasion in GBM. We first established U87 cells that stably expressed miR-211 and named these cells LV-miR-211, cells used as negative control were named LV-control (Figure 2A). The MTT assay revealed that LV-miR-211 cells grew more slowly than the LV-control cells (Figure 2B). The colony formation assay demonstrated that LV-miR-211 cells formed smaller and less colonies than the LV-control cells (Figure 2C). The boyden assay was used to determine the effect of miR-211 on cell invasion. It was found that cell invasion was significantly decreased in LV-miR-211 cells (Figure 2D).

**Figure 2:** Restoration of miR-211 inhibited GBM cell growth and invasion *in vitro* **A**. Cells were stably transfected with miR-211. **B**. LV-miR-211 cells grew slower than the LV-control cells. **C**. LV-miR-211 cells formed less and smaller colonies than the LV-control cells. **D**. The cell invasion ability was significantly decreased in LV-miR-211 cells.

### MiR-211 inhibited GBM cell stress fibre expression and reversed the EMT phenotype

Cytoskeletal reorganization, exemplified by the formation of stress fibre bundling arrays, is essential for the contractile motion of cancer cells [18]. With the use of phalloidin staining, we revealed that stress fibre formation was suppressed in LV-miR-211 cells when compared with LV-control cells (Supplementary Figure 1A). The EMT phenotype is considered to be a key regulator of cancer cell invasion [19]. By Western blot we found that the expression level of epithelial marker E-cadherin increased, while mesenchymal markers N-cadherin and Vimentin decreased in LV-miR-211 cells (Supplementary Figure 1B). Similar results were found by immunofluorescence assay (Supplementary Figure 1C).

### Restoration of miR-211 decreased cell growth and invasion *in vivo*

We next investigated the efficacy of miR-211 against tumor growth and invasion *in vivo*. When compared with LV-control cells, LV-miR-211 cells resulted in decreased growth and tumor weight of subcutaneous xenograft tumors in nude mice (Figure 3A and 3B). In the experimental metastasis studies, LV-miR-211 cells established smaller lung and liver metastatic colonies than the mock group (Figure 3C and 3D). These results suggest that miR-211 could inhibit the growth and metastasis of GBM cells *in vivo*.

**Figure 3:** Restoration of miR-211 decreased cell growth and invasion *in vivo* **A**. and **B**. LV-miR-211 cells resulted in decreased growth and tumor weight of subcutaneous xenograft tumors in nude mice. **C**. and **D**. LV-miR-211 cells established smaller lung and liver metastatic colonies than the mock group.

### HMGA2 was a direct target of miR-211 in GBM

Targetscan and miRanda algorithms were used to search for target genes of miR-211. From the mRNAs containing miR-211 recognition sites in their 3′-UTRs, we focused on HMGA2, which is associated with cancer cell proliferation and invasion. To examine if HMGA2 was a direct target of miR-211, HMGA2 wild-type (WT) or mutant 3′-UTR (Figure 4A) were subcloned into a luciferase reporter vector and co-transfected with miR-211 mimics or negative control into U87 cells. We revealed that miR-211 significantly inhibited the luciferase activity of the HMGA2 WT 3′-UTR but not of the mutant in U87 cells (Figure 4B). Subsequently, we transfected miR-211 into U87 cells and found that overexpression of miR-211 reduced the mRNA and protein levels of HMGA2 (Figure 4C and 4D). These findings indicate that HMGA2 is a direct downstream target for miR-211 in GBM cells.

**Figure 4:** HMGA2 was a direct target of miR-211 **A**. HMGA2 wild-type (WT) and mutant 3′-UTR as indicated. **B**. miR-211 significantly inhibited the luciferase activity of the HMGA2 WT 3′-UTR but not of the mutant in U87 and U251 cells. **C**. miR-211 reduced the mRNA level of HMGA2 in U87 and U251 cells. **D**. miR-211 reduced the protein level of HMGA2 in U87 and U251 cells.

We then asked whether restoration of HMGA2 could rescue the effects of miR-211 on cell growth and invasion. Transfection of pcDNA.3-HMGA2 into LV-miR-211 cells could increase the HMGA2 expression (Supplementary Figure 2A). In addition, transfection of HMGA2 into LV-miR-211 cells restored the decrease in proliferation and invasion induced by stable overexpression of miR-211 (Supplementary Figure 2B-2D). qRT-PCR was used to measure the relation between miR-211 expression and HMGA2 expression in GBM patient samples. We found that there was a negative association between miR-211 and HMGA2 expression (Supplementary Figure 2E, r=-0.763).

### Restoration of miR-211 inhibited the AKT/β-catenin pathway

To determine the downstream mechanisms underlying the role of HMGA2 in the tumor-suppressing effects of miR-211, we investigated the AKT/β-catenin signaling pathway. Restoration of miR-211 decreased p-AKT and nuclear β-catenin expression, whereas anti-miR-211 had the opposite effect (Figure 5A). Restoration of HMGA2 resulted in the recovery of p-AKT and β-catenin expression that had been weakened through transfection with miR-211 into glioma cells (Figure 5B). We also revealed that overexpression of miR-211 decreased nuclear β-catenin expression, while restoration of HMGA2 counteracted this effect, as determined by the immunofluorescence assay (Figure 5C).

**Figure 5:** miR-211 inhibited the AKT/β-catenin pathway **A**. Restoration of miR-211 decreased p-AKT and nuclear β-catenin expression, whereas anti-miR-211 had the opposite effect. **B**. Restoration of HMGA2 resulted in the recovery of p-AKT and nuclear β-catenin expression that had been weakened through transfection with miR-211. **C**. Overexpression of miR-211 inhibited nuclear β-catenin expression, while restoration of HMGA2 counteracted the effect.

### EZH2 repressed miR-211 expression through H3K27me3

We further asked whether the downregulation of miR-211 in GBM was due to methylation of its promoter region. Bisulfite sequencing PCR (BSP) revealed that the methylation of miR-211 was higher in GBM cell lines when compared with normal brain cells (Figure 6A). Subsequently, we examined H3K27me3 levels around the promoter region of miR-211 by performing chromatin immunoprecipitation (ChIP) assay. We observed that H3K27me3 was steadily enriched at the promoter region of miR-211 (Figure 6B). EZH2 downregulation or cells treated with deazaneplanocin A (DZNep) increased the levels of miR-211 (Figure 6C and 6D). These results support the notion that miR-211 is epigenetically silenced by DNA methylation and EZH2-mediated histone methylation in GBM.

**Figure 6:** EZH2 repressed miR-211 expression through H3K27me3 **A**. Hypermethylation of the miR-211 promoter was detected in GBM cell lines. A schematic distribution of CpG islands is illustrated by the vertical bars. At least two single clones are represented for each sample. Black and white circles represent hypermethylation and hypomethylation, respectively. **B**. Schematic representation of the miR-211 locus showing the relative positions of the ChIP PCR forward primers H3K27me3 was steadily enriched at the promoter region of miR-211. IgG was used as a control. **C**. EZH2 downregulation increased the expression of miR-211. **D**. DZNep treatment increased the expression of miR-211.

## DISCUSSION

MiRNAs contribute to the development and metastasis of GBM, and are suggested to be novel therapeutic targets for the treatment of GBM [20, 21]. Mounting evidence suggests that miR-211 inactivity is associated with multiple types of cancer. A previous study demonstrated that the expression level of miR-211 was decreased in glioma [22]. However, the effects and underlying molecular mechanisms of miR-211 in regulating GBM development are poorly understood. In the present study, we revealed that miR-211 was downregulated in GBM tissues and cell lines. Interestingly, GBM patients with high miR-211 expression had longer overall survival time than those with low miR-211 expression. These data suggest that miR-211 may be a tumor suppressor in GBM.

To verify our hypothesis, we re-introduced miR-211 into GBM cells. We revealed that restoration of miR-211 inhibited GBM cell proliferation and invasion both *in vitro* and *in vivo*. Deng et al. found that ectopic expression of miR-211 restricted hepatocellular carcinoma cell proliferation, migration and invasion both *in vitro* and *in vivo* [23]. In parallel, Xia et al. found that miR-211 suppressed epithelial ovarian cancer proliferation through affecting cell-cycle progression [12]. Our findings are similar to these observations and confirm that miR-211 functions as a tumor suppressor in GBM.

Subsequently, we identified HMGA2 as a direct target of miR-211. MiR-211 negatively regulated HMGA2 expression, as determined by luciferase reporter and Western blot assays. HMGA2 is an architectural transcription factor that plays a crucial role in the development and progression of various malignant cancers. Abnormal expression of HMGA2 usually promotes cancer cell proliferation and invasion [24]. In GBM, the decreased expression of HMGA2 promoted cell invasion and stemness [25, 26]. We observed that HMGA2 overexpression could rescue the effect of miR-211 on GBM cells. Interestingly, we found that there was a negative correlation between miR-211 and HMGA2 expression in GBM tissues. HMGA2 is able to activate the AKT signaling pathway [27]. AKT could lead to phosphorylation of β-catenin and promotes Wnt pathway signaling. AKT-mediated phosphorylation of β-catenin causes its disassociation from cell-cell contacts and its accumulation in both the cytosol and the nucleus. Phosphorylation of β-catenin by AKT increases its transcriptional activity and promotes tumor cell invasion [28]. The Wnt canonical pathway can active nuclear β-catenin. When the Wnt signal is absent, free cytoplasmic β-catenin is phosphorylated by serine/threonine kinases and GSK3β in a large APC/axin scaffolding complex that targets β-catenin for degradation. When the Wnt signaling is present, this destruction complex is disrupted, and dissociation of GSK3β prevents phosphorylation of β-catenin. The Wnt signial can increase the stability of β-catenin and lead to its translocation in the nucleus [29, 30]. However, β-catenin can also be activated by the non-canonical pathway [31]. The abnormal expression of microRNAs often contribute to the activation of β-catenin [32, 33]. Our study found that miR-211 could inhibit the activation of the AKT/β-catenin signaling pathway through negatively regulating HMGA2. We thus propose that the effects of miR-211 on GBM cell proliferation and invasion is mediated by the HMGA2/AKT/ β-catenin axis.

Furthermore, our study revealed that the dysregulation of miR-211 was caused by promoter methylation. Polycomb repressor complex 2, of which EZH2 is the catalytic component, mediates trimethylation of histone 3 at lysine K27 (H3K27) and subsequent repression of target genes [34]. EZH2 is frequently over-expressed in cancer and contributes to miRNAs silencing. For instance, EZH2 suppresses miR-31 expression by inducing H3K27me3 on the miR-31 promoter in prostate cancer [35]. In hepatocellular carcinoma, miR-622 is transcriptionally repressed by EZH2-induced H3K27 trimethylation and promoter methylation [36]. These results support the role of EZH2 in miRNA downregulation during cancer progression. In parallel, our findings revealed that EZH2 suppressed miR-211 expression through H3K27 trimethylation. To the best of our knowledge, this is the first report which demonstrates the role of the EZH2/miR-211/HMGA2/AKT/β-catenin axis in GBM progression.

Taken together, our results provide evidence that miR-211 is involved in the development of GBM. Furthermore, we demonstrated that miR-211 functions as a tumor suppressor in GBM, at least, partly through repression of the HMGA2/AKT/β-catenin axis. In all, our findings suggest that miR-211 could be a potential target in the treatment of GBM.

## MATERIALS AND METHODS

### Cell lines culture and patient samples

Human GBM cell lines (SWO-38, U251, U87 and U211) were cultured in a humid atmosphere containing 5% CO_2_ at 37°C in RPMI-1640 medium supplemented with 10% fetal bovine serum, 100 U/mL penicillin, and 100 mg/mL streptomycin. Cell lines were purchased from the Institute of Biochemistry and Cell Biology of the Chinese Academy of Sciences (Shanghai, China). GBM patient samples were obtained from the Affiliated Cancer Hospital of Guangzhou Medical University. Normal brain cells were cultured as previously described [37]. This study was conducted with the approval of the Ethical of Guangzhou Medical University.

### Lentivirus production and infection

The pLV-has-miR-211 plasmid and the negative control pLV-miRNA-vector were purchased from Biosettia Inc. (San Diego, USA). Viral packaging and infection were performed according to standard protocols as recommended by the manufacturer. The packaged lentiviruses were named LV-miR-211 and LV-control accordingly.

### Cell transfection

MiR-211 mimics and the negative control miR-ctrl were synthesised by Genepharma (Shanghai, China). Oligonucleotide transfection was performed with Lipofectamine 2000 reagent (Invitrogen) according to manufacturer's instructions.

### Dual luciferase activity assay

Full-length HMGA2 cDNA lacking the 3′-UTR was subcloned into the eukaryotic expression vector pcDNA3 (+) (Invitrogen). The HMGA2 3′UTR target site for miR-211 was amplified by PCR and cloned into the XbaI site of pGL3 control (Promega, Madison, USA). This vector was sequenced and named WT HMGA2 3′UTR. Site-directed mutagenesis of the miR-211 target-site in the HMGA2 3′UTR was carried out using the Quick-change mutagenesis kit (Stratagene, Heidelberg, Germany) and named Mut HMGA2 3′UTR. For the reporter assays, Wt or Mut HMGA2 3′UTR vector and the control vector pRL-CMV ((cytomegalovirus) coding for Renilla luciferase, Promega) were cotransfected. Luciferase activity was measured 24 hours after transfection using the Dual-Luciferase Reporter Assay System (Promega).

### Q-RT-PCR and western blot assays

We extractedtotal RNA with the use of TRIzol reagent (Invitrogen). To detect miR-211, qRT-PCR reactions were performed using the standard SYBR Green Assay protocol and the ABI PRISM 7500 Sequence Detection System (ABI). The primers for miR-211 were 5′-GCTCGTCGGGTCGGGCCTATTG-3′ (forward) and 5′-CCGCCCCTATTGCTTAAGCCCACG-3′ (reverse). U6 snRNA was used as a normalization control. qRT-PCR analysis for HMGA2 and the normalization control gene GAPDH were performed using SYBR Premix Ex Taq (TaKaRa, Dalian, China). The primers for HMGA2 were 5′-TACCCCTGGAGCCGCGGGC-3′ (forward) and 5′-CTGGGACGTCAGACCCTG-3′ (reverse). The primers for GAPDH were 5′-AACGTGTCAGTGGTGGACCTG-3′ (forward) and 5′-AGTGGGTGTCGCTGTTGAAGT-3′ (reverse). The relative expression of each gene was calculated and normalized to U6 snRNA or GAPDH using the 2^−ΔΔCt^ method.

For western blot assay, equal amounts of protein were resolved by SDS-PAGE and transferred to a polyvinylidene fluoride (PVDF) membrane. Subsequently, the membranes were blocked in 5% BSA, followed by protein detection with primary antibodies at 4°C overnight. After washing with TBSA, the proteins were detected with appropriate secondary antibodies.

### MTT assay, colony assay, boyden assay and in situ detection of miR-211

The MTT assay was carried out as previously described [38]. For the cell invasion assay, cells (1×10^6^) were placed into chambers which were coated with 150 mg of Matrigel (BD Biosciences, Boston, MA, USA). The chambers were inserted into the wells of a 24-well plate and incubated for 36 hour in RPMI-1640 medium supplemented with 10% fetal bovine serum. The cells remaining on the upper surface of the membrane were removed, and the cells adhering to the lower surface were fixed, stained in a dye solution containing 0.05% crystal violet and counted. In situ detection of miR-211 in paraffin-embedded GBM tissue and normal brain samples was carried out as previously described [39].

### *In vivo* tumor growth and invasion assay

All procedures involving animals were approved by the Institutional Committee on Animal care, Guangzhou Medical University. Cells were mixed with growth factor-reduced phenol red-free Matrigel and injected subcutaneously into both flanks of nude mice. Four weeks later the xenografts were removed from the mice and weighed. Tumor volume was calculated using the following formula: 4π/3 × (width/2)^2^ × (length/2).

The invasion assay was carried out as previously described [40]. Briefly, mice received a single intravenous tail vein injection of 10^6^ cells. Six weeks later, the mice were sacrificed. Subsequently, individual organs were removed and metastatic tissue was analyzed using hematoxylin and eosin (H & E) and immunohistochemical (IHC) staining.

### DNA methylation analysis

Bisulfite conversion was carried out using 1 mg of DNA using an Epitect Bisulfite Kit (Qiagen). Bisulfite-treated DNA was amplified with BSP primers located in the miR-211 promoter region: 5′-GTTATTGAAGTTAATAACGGTGATTGATA-3′ (forward) and 5′-CTTCCTCGGAATTAACTATTACTGCG-3′ (reverse).

### Chromatin immunoprecipitation assay

CHIP assay was performed using the EZ-CHIP chromatin immunoprecipitation kit (Millipore, Billerica, MA) according to the manufacturer's protocol. Captured genomic DNA was obtained and used for quantitative PCR analysis. The primers used for detection of the miR-211 promoter sequence were as follows: P1 5′-CTTGCAGGTTCCAGAGGAGA-3′ (forward) and 5′-CGAGTCTTGGGCTCGGAA-3′ (reverse); P2 5′-GCCCACAGGTTTGAAGGAC-3′ (forward) and 5′-CGGGATAGCAAGACATTTGG-3′ (reverse); P3 5′-CGGGAAGTCATGAACCTACC-3′ (forward) and 5′-GCGGACCATGGGTAATGGAT-3′ (reverse); P4 5′-CCGGGAATAAACAGATAAAG-3′ (forward) and 5′-TTGGTGGGCGACAAACC-3′ (reverse).

### Statistical analysis

SPSS 13.0 and Graph Pad Prism 5.0 software were used for statistical analysis. All values are presented as mean values ± S.E.M. One-way ANOVA or two-tailed Student's t-test was used for comparisons between groups. The relationship between HMGA2 and miR-211 expression was explored by Spearman's correlation. A P value of <0.05 was considered statistically significant.

## SUPPLEMENTARY FIGURES


